The article "Bioactivity of Exosomes Derived from Trained Natural Killer Cells versus Non-Trained One: More Functional and Antitumor Activity" was published in 2022. Journal: Biomed Res Int.

# Bioactivity of Exosomes Derived from Trained Natural Killer Cells versus Non-Trained One: More Functional and Antitumor Activity

**DOI:** 10.1155/2022/5396628

**Published:** 2022-08-24

**Authors:** Fateme Mohammadi, Zahra Sadat Hashemi, Ramin Sarrami Forooshani, Shaban Alizadeh

**Affiliations:** ^1^Department of Hematology, School of Allied Medical Sciences, Tehran University of Medical Sciences, Tehran, Iran; ^2^ATMP Department, Breast Cancer Research Center, Motamed Cancer Institute, ACECR, Tehran, Iran

## Abstract

**Background:**

Natural killer (NK) cells are cytotoxic lymphocytes of the innate immune system, capable of killing viral-infected and cancerous cells. NK cell-mediated immunotherapy has remarkably changed the current paradigm of cancer treatment in recent years. It emerged as a safe and effective therapeutic approach for patients with advanced-stage leukemia. Several immune-escape mechanisms can be enacted by cancer cells to avoid NK-mediated killing. Exosomes released by NK cells that carry proteins and miRNAs can exert an antitumor effect. In the present study, we hypothesized that maybe exosomes derived from trained natural killer cells show more antitumor effect in comparison to non-trained one.

**Methods:**

PBMC was separated by the Ficoll method and cultured with IL-2 for 21 days to expand NK cells. The NK cells were co-cultured with K562 for 72 hours and exosome-derived co-cultured (as trained) and natural killer cell-derived exosomes (as non-trained) were extracted by Exo kit. The exosomes were confirmed by dynamic light scattering (DLS), transmission electron microscopy (TEM), flow cytometry, and western blotting. The K562 cells were separately treated by trained and non-trained exosomes and MTT assay, apoptosis, and real-time PCR were performed.

**Results:**

Based on flow cytometry, CD56 marker was 89.7% and 40.1% for NK cells and NK-derived exosomes, respectively. CD63 and CD9 were positive for exosomes by western blotting. The morphology of exosome was confirmed by TEM. Treated K562 cells by trained exosomes indicated the diminished cell viability and higher apoptosis. Furthermore, the trained exosomes showed up-regulation in both P53 and caspase3 genes as compared with non-trained sample. *Discussion*. Trained Exos showed a potent inhibitory effect on proliferation and induced apoptosis on K562 cell lines compared to the same dose of non-trained Exos. According to the results of qRT-PCR, trained Exos exerted an antitumor activity through up-regulation of caspase 3 and P53 in the apoptotic signaling pathway in tumor cells. Our findings indicate an effective action of trained Exos against cancer cells.

## 1. Introduction

Cancer is one of the main causes of death in the world, and different types of treatments were performed for cancer therapy to decrease the number of deaths. Resembling the radiation therapy targets all cells localized in the tumor microenvironment, and chemotherapy sets a goal on all rapidly growing and dividing cells. However, both of them are traditional cancer therapy. Actually, in these methods, not only cancer cells, even normal cells, are subjected which can even lead to the escape of cancer cells from traditional therapy methods [1]. Also, side effects such as pain, nausea, diarrhea, cardiotoxicity, and hair loss are another problem of these treatments [2]. The new generation of treatment was based on immunotherapy [3]. Nowadays, cancer immunotherapy is one of the hot topic challenges in the sciences [4]. Two astounding classes of cancer immune cell therapy are natural killer (NK) cells and CAR-T cells. However, CAR-T cells therapy can trigger cytokine storm and stem cell transplantation [5–7] can cause graft-versus-host disease, but NK cell therapy does not have which leads to low risk of NK cell immunotherapy for patients [8].

NK cells develop from lymphoid progenitor cells in the bone marrow [9] and are about 10-15% of total lymphocytes in peripheral blood. NK cell surface marker is CD3^−^CD56^+^ that is recognized in two subtypes, CD56^bright^CD16^dim^: the immature form of NK cells with 10% of whole NK cells, and CD56^dim^CD16^bright^: the mature NK cells [10]. The cytotoxicity functions of NK cells are against the damaged, infected, and/or pre-malignant cells in the innate immune system [11]. Their cytotoxicity can be regulated by effector molecules such as interferon (IFN-*γ*), tumor necrosis factor (TNF-*α*), and interleukin (IL) 2, 12, 15, and 18 [12]. Actually, the immature form of NK cells is responsible for cytokine production (INF-*γ*), and mature NK cells' function has stored granzymes and perforin [13]. NK cells showed therapeutic potential for human leukemia and other malignancies [14]. IFN-*γ* is produced by immune cells in response to microbial pathogens [15]. NK cells can be influenced by the hypoxic and acidic environment of a tumor so the tumor cells could be escaped from these killer cells, but these environments cannot affect extravascular (EVs) which were secreted by NK cells [16, 17].

Extravascular (EVs) are lipid bilayer vesicles which are released by most cells. Their size is about 50-1000 nm and can be found in body fluids such as blood, saliva, urine, and breast milk [18]. EVs can be classified into apoptotic bodies, microvesicles, and exosomes. This classification is based on their size, morphology, biogenesis, and phenotype [19]. The exosomes are small EVs, whose size is about 50-150 nm, and their morphology is cup-shaped which is recognized by transmission electron microscopy (TEM). The exosomes' common membrane markers are CD63, CD81, CD9, and some proteins that are involved in vesicular trafficking such as Alix and tsg101 [20]. Several studies have shown that exosome-derived NK cells contain FasL, perforin, granzyme A, B, granulysin, proteins, microRNAs [21–23], other non-coding RNA, and mRNA, and the same as their parental cells (NK cells) [24–26]. It seems that exosome-derived NK cells which contain several biomolecules have various biological activity, such as antitumor effect. And activity status of NK cells may effect on the nature and function of these exosomes.

In this study, we have shown the difference in the bioactivity of exosome-derived NK cells pre-exposed to CML cells and the exosomes derived from intact NK cells in the induction of tumor cell death. This is the first time that pre-contact exosomes with cancer cells were used for killing cancer cells. Our goal in this study was to determine the efficacy of trained exosomes on the killing activity on b CML cells compared to non-trained exosomes.

## 2. Method and Material

### 2.1. NK Cell Isolation and Expansion

From a healthy donor, 30 ml heparinized blood samples were drawn and after dilution in PBS buffer, the suspension was loaded on Ficoll (Ficoll-solution, GE Health care-Sweden) and centrifuged at 800 × g for 30 min. Then, PBMCs were collected from the buffy coat layer and washed twice with PBS [27]. For expansion and activation of NK cells, isolated PBMCs were cultured with the following components: 6 ml of RPMI1640 (Gibco-USA), 1000 IU/ml recombinant human IL-2 (Miltenyi Biotec-USA), 10 ng/ml OCT3 (Miltenyi Biotec-USA), and 5% autologous human plasma into untreated T25 flasks. The conditioned medium containing 500 IU/ml rhIL-2 was added every three days until day 21. Expanded cells were transferred into new flasks. Viability was determined with 4% trypan blue exclusion dye (Sigma-USA) before each experiment. Cells with viability less than 98% were excluded from the study.

#### 2.1.1. Flow Cytometry Analysis of NK Cells

The specific surface markers were used to detect the purity of the expanded NK cells. Indeed, the PBMCs were analyzed by flow cytometry immediately after collecting blood from a donor, whereas NK cells were examined after 21 days of culturing. Though two experiments were performed on different days, we used the same flow cytometry conditions such as compensation, threshold, gating, and cell numbers to minimize possible technical variations between the two experiments. The cell suspension was incubated by 1 *μ*g FITC-labeled anti-CD3 and 1 *μ*g PE-labeled anti-CD56 (Biolegend-USA) in 100 *μ*l PBS (Sigma-Germany) containing 2% human albumin (Sigma-Germany) for 30 min at 4°C. Finally, cells were washed by PBS and read on Attune NxT flow cytometry.

### 2.2. Cell Culture

K562 cell lines are one of the CML types taken from a patient with CML [28]. This cell line was received from Motamed Cancer Institute (Tehran, Iran) and maintained in RPMI-1640 supplemented with 5% FBS (fetal bovine serum) and 1% penicillin/streptomycin, and grown in 5% CO_2_ at 37°C. The K562 cells (5 × 10^5^) and NK cells (5 × 10^6^) co-cultured (NK-K562) in RPMI-1640 supplemented by 5% exosome-depleted FBS for 72 hours (exosome-depleted FBS as the exosome-free serum was prepared by centrifugation at 4,000 g for 10 min with a 100 kDa Amicon filter (Merck Millipore)).

### 2.3. Exosome Isolation

The NK cells (5 × 10^6^) and NK-K562 cells were cultured for 3 days in T25 cell culture flask. Consequently, the total medium of each group (nearly 15 ml) was collected. The exosomes from the supernatant of intact NK (as non-trained Exos) and from the NK-K562 media (as trained Exos) were purified using the Exo-spin kit (Cell Guidance Systems) according to the manufacturer's instruction. In brief, the cell culture medium was centrifuged at 16,000 g for 30 min to remove any remaining cell debris. The supernatant was transferred to a new tube without disturbing the pellet, mixed with the kit buffer, mix the culture media/reagent by vortexing, and incubated overnight at 4°C. After incubation, the samples were centrifuged at 10000 g for 1 hour at 4°C. The pellet was suspended in PBS, and for further purification, it was applied to the top of the column. Isolated exosomes were stored at -70°C until use.

### 2.4. Exosome Characterization

#### 2.4.1. Measurement of Concentration

The isolated exosome concentration was determined by Bradford test. Briefly, 2 *μ*l of protein (isolated exosome) was diluted in buffer (total volume was about 50 *μ*l). After that, 50 *μ*l of Coomassie reagent was added to the diluted samples in a 96-well plate. The absorbance of the mixture was determined at 592 nm with a microplate reader, and the protein concentration was estimated. A calibration curve was constructed using bovine serum albumin as a protein standard exactly according to the protocol which is described above.

#### 2.4.2. Measurement of Particle Size and Zeta Potential

Dynamic light scattering (DLS) system (HORIBA-SZ100 Instruments) was used for exosome particle size analysis, and Zeta potential measurements were performed using the ZS100 (HORIBA). 10 *μ*g of exosomes was diluted in PBS and analyzed three times before examination. Actually, the size distribution was determined by signal intensity and Z-average diameter obtained from autocorrelation function using general-purpose mode.

#### 2.4.3. Transmission Electron Microscopy (TEM)

The exosome's morphology was studied by TEM. Approximately 200 *μ*l of exosomes was dropped onto the formvar/carbon-copper grid, Mesh300. After 1 min, excess water was removed by touching the grid with a piece of filter paper. The material on each grid was fixed with 2% phosphotungstic acid (PTA) for 10 min, rinsed with deionized water, and negatively stained with 1% uranyl acetate for 15 min to remove the negative background. After drying, the copper nets were examined with PLILIPs, EM208S TEM (NETHERLAND) at 100 kV.

#### 2.4.4. Exosome Flow Cytometry

To characterize the isolated exosomes, a biotinylated anti-CD56 antibody (eBiosciences-USA) labeled by PE (phycoerythrin) was used to detect the CD56-positive exosomes. Raw data were then analyzed using conventional Flowjo™ 10.8 software.

#### 2.4.5. Western Blot

Total NK cell-derived exosomes (10 *μ*g) were separated on a 12.5% sodium dodecyl sulfate-polyacrylamide gel electrophoresis (SDS-PAGE) and transferred to nitrocellulose transfer membranes (PROTRAN, Schleicher & Schuell BioScience, Germany). The membranes were blocked with 3% skim milk in Tris-buffered saline/0.05% Tween-20 (TBS-T) for 1 hour and then incubated with freshly prepared primary antibody solutions: anti-CD9, CD63, and calnexin at a dilution of 1 : 1000 overnight at 4°C. After washing with TBS-T, the secondary antibody IRDye 680RD (Licor) was added at a dilution of 1 : 10,000 for 1 hour at room temperature. The band was visualized by scanning both 700 and 800 nm channels of the LI-COR Odyssey infrared imaging system.

### 2.5. Evaluation of Cancer Targeting

#### 2.5.1. Cell Uptake Assay

Exosomes were labeled with PKH26 red fluorescent lipid membrane dye (Sigma-Aldrich, USA). 60 *μ*l PKH26 dye was diluted in 60 *μ*l diluent C (dye solution). Then, 30 *μ*g of exosomes wereadded to the dye solution and incubated for 15 min at room temperature. After incubation, 120 *μ*l BSA 1% was added to exosomes and dye solution, then transferred to 100 kDa Amicon column and centrifuged at 400 × *g* for 1 min at 4°C. The exosomes were washed three times with 1 ml PBS before being concentrated to a final volume of 50 *μ*l. K562 cells was treated by PKH26 labeled exosomes then visualized with an inverted fluorescence microscope.

#### 2.5.2. Cell Viability

K562 cancer cell lines were seeded at a density of 2x10^4^ cells/well in a 96-well plate. After that, the trained and non-trained Exos were applied to the wells with different concentrations (1, 3, 5, 7, and 10 *μ*g/well). After 48 hours, 10 *μ*l of methyl thiazolyl tetrazolium (MTT, 5 mg/ml in PBS; Sigma, St Louis, Missouri) was added for 4 hours at 37°C in a 5% CO2 incubator. Formazan crystals were resolved with mixture of SDS and sulfuric acid (about 100 *μ*l/well). The OD at a wavelength of 570 nm was measured with a spectrophotometer. Half maximum inhibitory concentration (IC50) was calculated for trained and non-trained Exo.

#### 2.5.3. Apoptosis Assay

Apoptosis was determined using the Annexin-V-FLUOS Staining Kit (Roche, Germany) according to the manufacturer's instruction. K562 cells were treated with trained and non-trained Exos for 48 hours. After that, the cells were harvested and resuspended in 100 *μ*l of incubation buffer followed by 2 *μ*l cocktail of Annexin-V fluorescein and propidium iodide (PI). After 15 min of incubation, the samples were analyzed by flow cytometry.

#### 2.5.4. Real-Time PCR

Total RNA was extracted using the RNeasy kit (FAVORGEN kit). The cDNA was primed from total RNA using the RevertAid First Strand cDNA Synthesis Kit (Fermentas, Thermo Fisher Scientific, and Waltham, MA). Real-time PCR assay was performed with the FastStartt SYBR Green MasterMix (Roche) on the ABI-7500 real-time PCR. All mRNA quantification data were normalized to *β*-actin, and the comparative Ct method (Pfaffl) was used to determine the expression fold change.

### 2.6. Statistical Analysis

All experiments were performed at least three times in triplicates for each group, and the SPSS software was used for data processing. Statistical significance was determined using Student's *t-*test and an asterisk means significant (*P* < 0.05).

## 3. Result

### 3.1. NK Cell Expansion and Characterization of Isolated Exosomes

The final count of NK cells after 21 days cultured with IL-2 cytokine was about 10^7^ cells/15 ml. NK cell colony and morphology were shown after 3 weeks (Figure 1(a)). The immune phenotyping of cells showed 89.7% CD56 positive population and 6.93% double-positive population for CD56 and CD3 (Figure 1(b)).

### 3.2. Characterization of Non-Trained and Trained Exosomes

NK and NK-K562 culture supernatants were harvested to isolate the exosomes using the Exo-spin kit. The exosome morphology as a spherical lipid bilayer vesicle for non-trained (Figure 2(a)), and trained Exos, was confirmed by TEM (Figure 2(b)).

The size distribution and Zeta potential of these lipid bilayer particles were obtained as 142.5 nm and -2.3 mV for non-trained (Figure 2(c)), and as 136.0 nm and -3.1 mV for trained (Figure 2(d)), respectively. The analytical technique for protein levels showed the positive expression of CD63 and CD9 specific markers in both non-trained and trained Exos. Notwithstanding, the calnexin (exosomal negative marker) was not detected in western blot (Figure 2(e)).

The heterogeneity of trained Exos (which contained exosomes derived both K562 and NK population) was analyzed by flow cytometry against CD56 marker. The expression of CD56, as the specific markers on the NK-derived exosomes, was measured by an anti-CD56 antibody conjugated to PE which indicated 34.9% for trained Exo compared to 41.0% for non-trained Exo (Figures 2(f) and 2(g)).

### 3.3. K562 Cells Treated by Exosomes

#### 3.3.1. Uptake of NK-Derived Exosomes

K562 cells were seeded in a 24-well plate, and 25 *μ*g of PKH26 labeled exosomes was added to each well. After 24 hours, cells were washed with PBS followed by visualization with an inverted fluorescence microscope (Figure 3(a)) and illustrated the uptake of NK-derived exosomes into the cell membranes of K562. The fluorescent intensity due to the presence of red PKH26 color demonstrated the existence of exosomes.

#### 3.3.2. Trained Exosomes Decreased the Cell Viability Efficiently

IC50 values were assessed 5.29 *μ*g/well for non-trained Exos and 4.13 *μ*g/well for trained Exos (Figures 3(b) and 3(c)). The K562 cells were divided into three groups: untreated, treated with 5.29 *μ*g/well of non-trained Exos, and treated with 5.29 *μ*g/well of trained Exos. All two treated groups showed the cytotoxic effects on the cells. However, the trained treated group significantly decreased the viability of cells at the same exosome concentration compared to the non-trained treatment group (*P* < 0.05) (Figure 3(d)).

#### 3.3.3. Apoptosis Assay

To further explore the effect of trained and non-trained Exos on K562 cell functions, trained and non-trained Exos in 5.29 *μ*g/well concentration were administrated in K562 cells. The apoptosis percentage was detected by Annexin V-PI which confirmed the cell apoptosis rate at 48 hours. The trained treated group illustrated 31.8% (early: 3.8 + late 28.0%) compared with control group (*P* < 0.05) (Figures 4(a) and 4(b)). The cytotoxicity of trained exosomes made the non-trained exosomes seem inconsequential by contrast.

#### 3.3.4. Real-Time PCR

The results of real-time PCR in (Figure 4(c)) showed that caspase 3 gene expression was increased in the treated groups more than control cells. On the other hand, the trained treated group indicated stunningly upper-expression compared to the non-trained group. P53 gene expression was up-regulated in all treated groups than the control group, but this increase was more in the trained exosomes group.

## 4. Discussion

K562 cell lines are used as a sensitive target cell and are widely used to assess in vitro NK cell function [29, 30]. The innate immune system is the first line defense against cancer and infections. Tumors can develop different mechanisms to evade the immune responses resulting in cancer growth and spreading. NK cells, as part of the innate immune system, contribute to tumor cell recognition and killing [31]. Lugini and colleagues showed that isolated NK cells from healthy donors were able to kill a variety of cancer cells [32]. Alicit et al. expanded NK cells by adding OKT3 (anti-CD3 antibody) in peripheral blood mononuclear cells (PBMCs) for the first 5 days, and also IL-2 (as the specific cytokine) for the remaining days. They did not use feeder cells and expanded NK cells had good quality and cytotoxicity function [33]. As well as in another study conducted by Di-Pace et al., it has been described that the stimulation of NK cells could be more effective by IL-2 or IL-15 cytokines [34]. This is consistent with our data, which OKT3 and IL-2 were used as supplements for NK cell expansion which resulting in 89.7% CD56 positive by flow cytometry.

The pharmaceuticals that were used in cancer therapy can be classified as small chemicals, macromolecules (protein, antibody, etc.), even though cells, and organs. These classifications depend on heterogeneity, functionality, and size of cancer tumors [35]. On the other hand, these materials have harshly side effects that caused the scientists turned to using safe carriers without side effects. During the past few years, one of the most beneficial carriers is liposomes. Indeed, liposomes can apply in drug targeting therapy, effectively. But the only downside of them was that it belongs to their artificiality fabrication. The fascinating thing about exosomes is it belongs to their natural essence while can be used as carriers (an alternative of liposomes), too. Their ability to be loaded with drugs, microRNA, or siRNA, their stability in peripheral blood, and their delivery to tumor sites are the attention results for exosome [31]. More than one trillion exosomes can be found in the peripheral blood injected into the patients in the blood transfusion of the clinical treatment. Namet al. suggested that exosomes administrated to the body in blood transfusion did not need matching for Human Leukocyte Antigen (HLA) and showed no immune-related reactions in the body [35]. Fabbri showed that NK-derived exsosomes had the cytotoxic effects against cancer cells. It can be occurred by granzyme A, granzyme B, granulysin, and perforin as exosomal cargo [32]. Perforin which secreted by NK-Exos is a pore-forming protein that can be directly inserted into the targeted cells [36, 37]. Consistent with the other experiments, in our experiment, K562 cell viability showed that NK-derived exsosomes account for the toxicity against the cancer cells.

Previous studies affirmed that CD56 as NK surface marker can also be used to isolate NK-derived exosomes [32, 38]. For this reason, the CD56 marker was detected for non-trained and trained exosome by flow cytometry after 3 days of NK culture and NK-K562 co-culture. Data values were assessed 34.9% for trained and slightly more for non-trained: 40.8%. This dissimilar percentage could be due to the simultaneous culture of cells in different population (NK cells and K562 cells in ratio 10 to 1). Choi et al. stated that NK cell cytotoxicity against K562 at ratio of 10 to 1 after 1 day was about 20% and after 7 days was about 70% [39].

Exoquick reagents are able to react with each other to form a mesh-like polymeric web that captures exosomes in a certain size (usually between 60 and 180 nm in diameter), which has been shown by Yuet al. This method is fast, simple, and requires only a low speed centrifuge [40]. The isolated NK-derived exosome size was measured about 124.8 ± 3.8 nm by Federici et al. [38]. In the current study, the exosomes were also extracted from intact NK cell culture supernatant by Exoquick reagent. Their size and Zeta potential have been measured by DLS: the size and Zeta potential were about 142.5 nm and -3.1 mV for non-trained Exos, respectively. On the other hand, the trained Exos Zeta and size were about -2.3 mV and 136.0 nm. These data showed that trained Exos did not show any significant difference with non-trained Exos. The most common exosomal surface markers are CD63, CD8, and CD9 [41, 42]. The CD63 and CD9 were positive markers that were also confirmed by western blot.

Beer, L et al. extracted exosomes from PBMCs, their qualitatively analyzed was performed by TEM. TEM images confirmed the typical size and shape of exosomes [43]. In our study, the exosome's shape and size were also approved by TEM. As Jung reported, exosomes are lipid bilayer cup-shape vesicles which visualized by negative stained TEM [44]. Here, no significant differences in morphology and physical characteristics were observed between non-trained Exos and trained Exos. Since the nature of exosome is considered a protein, the conventional quantification method can be used. As in Beer's study, exosomal concentration was measured by Bradford [43]. Our investigation illustrated 315 *μ*g non-trained Exos and 196 *μ*g trained Exos isolated in total. Di et al. showed that pure NK-derived exosomes can exert rapidly cytotoxic activity on targets cells even at low concentrations, more than intact NK cells [34]. It has been demonstrated that the cytotoxicity property of NK-Exos depends on the dose and the duration exosomal treatment [45]. Some studies reported that NK-Exos efficiently killed tumor cells, while their cytotoxic consequence was reduced against non-tumor cells [34]. Apoptosis induction as an important mechanism in NK cell-based immunotherapy caused cellular toxicity. As described previously, perforin is one of the NK-Exos cargo which can stimulate the intrinsic apoptotic pathway and increase the release of cytochrome C, although FasL (which expressed on the membrane of NK c ell-released exosomes) can trigger the extrinsic pathway by activating caspase 8 and 3 [46]. The cytochrome C is released from mitochondria that activate caspase 9, which consequently stimulated caspase 3 and 7. Hence, the apoptotic pathway was stunningly occurred in NK-Exos treated cells [47, 48]. Han, D et al. showed that caspase 3 mRNA expression was increased in NK-Exos treated cell [49]. In our report, NK-derived exosomes can evaluate apoptosis in treated cells; it shows that cells treated with trained exosomes can induce more apoptosis compared with non-trained exosomal treated cells. In addition, real-time PCR confirmed that caspase 3 and P53 (plays a major role in apoptosis) gene expressions had up-regulated in trained and non-trained exosomal treated groups, although trained exosomal treated groups had more gene expression in both P53 and caspase 3 than non-trained one.

It seems that training NK cells with a target cell may change the composition of exosomes which became more bioactive in the immunologic functions and show more cell cytotoxicity effect on tumor cells.

In conclusion, the trained Exos have unique properties and anticancer activity that make them promising candidate agents for cancer immunotherapy. In a way, trained Exos contain a memory of dealing with the cancer cell, which causes them to show severe cytotoxicity in re-exposure versus the cancer cell. Therefore, exosome-derived NK cells obtained through cancer patients showed an intense reaction in a new encounter with the cancer cell. These can be collected, *ex vivo* expanded, and followed by administration as cellular products therapy. Besides, exosomes from natural killer cells that have been expanded by a feeder cell (K562) can also be more lethal. To our knowledge, this is the first report to demonstrate the more antitumor effect of trained Exos; however, further *in vivo* studies are needed to clarify whether this inhibitory effect is due to the increased cellular concentrations of anticancer signaling molecules as the exosome's cargo or the memorial antitumor effect of NK-Exos.

## Figures and Tables

**Figure 1:** NK cell expansion. NK cell morphology in colony expansion (a). NK cell purity in the case of CD3 and CD56 expression after 21 days in specific media (b).

**Figure 2:** Exosome characterization. The exosome morphology as a spherical lipid bilayer vesicle for non-trained (a) and trained Exos (b) was confirmed by TEM. The size distribution and Zeta potential were obtained as 142.5 nm and -2.3 mV for non-trained Exos (c) and as 136.0 nm and -3.1 mV for trained Exos (d). The positive expression of CD9 and CD63, the general Exos markers, and non-expression of calnexin were analyzed by western blot (e). The expression of NK-Exos specific proteins (CD56) was analyzed by using flow cytometry for non-trained Exos (f) and trained Exos (g).

**Figure 3:** Cytotoxicity of trained Exos compared to non-trained Exos. K562 cells were seeded in a 24-well plate, and 25 *μ*g of PKH26 labeled exosomes was added to each well. The red fluorescent was visualized by an inverted fluorescence microscope. The fluorescent intensity due to the presence of red PKH26 color demonstrated the existence of exosomes (a). IC50 values were assessed 5.29 *μ*g/well for non-trained Exos (b) and 4.13 *μ*/well for trained Exos (c). The K562 cells were divided into three groups: untreated, treated with 5.29 *μ*g/well of non-trained Exos, and treated with 5.29 *μ*g/well of trained Exos. The cell viability was confirmed by MTT after 48 hours (d). Data are presented as means ± SD of three separate experiments, *n* =3, ∗*P* < 0.05 vs control groups.

**Figure 4:** The effect of trained Exos on the cell apoptosis and gene expression. (a) The apoptosis percentage of K562 cells was detected by Annexin V-PI using flow cytometry which confirmed the cell apoptosis rate at 48 hours (Q1: Necrosis, Q2: Late Apoptosis, Q3: Early Apoptosis, Q4: Live Cells). (b) Data (Late and Early Apoptosis) are presented as means ± SD of three separate experiments, *n* =3, ∗*P* < 0.05 vs control group. The trained treated group illustrated 31.8% (early: 3.8 + late 28.0%). (c) The expression levels of P53 and caspase 3 genes were examined in treated groups compared to the control groups by real-time PCR (Pfaffl ratio) and normalized to *β*-actin expression level. Caspase 3 and P53 gene expression were increased in all treated groups more than control cells. On the other hand, the trained treated group indicated stunningly upper-expression compared to the non-trained group (g). Data are presented as means ± SD of three separate experiments, *n* =3, ∗*P* < 0.05 vs control groups.

## Data Availability

The authors can also make data available on request through a data access committee, institutional review board, or the authors themselves.
